The article "Deconstruction of the Optimal Design of Urban Road Interchange Based on the Integration of Smart Transportation and Big Data" was retracted in 2023. Reasons: unreliable results or conclusions; concerns about the data; concerns about the peer review; concerns about the citations.

# Deconstruction of the Optimal Design of Urban Road Interchange Based on the Integration of Smart Transportation and Big Data

**DOI:** 10.1155/2022/4241097

**Published:** 2022-08-13

**Authors:** Jiyong Zhang, Yukui Yang, Lijing Chu, Shiliang Chen, Wenchao Bian, Meining Ling, Shengfu Li

**Affiliations:** ^1^Guangzhou Urban Planning & Design Survey Research Institute, Guangzhou, Guangdong 510060, China; ^2^Guangdong Enterprise Key Laboratory for Urban Sensing, Monitoring and Early Warning, Guangzhou, Guangdong 510060, China; ^3^Production & Technology Department, Guangzhou Municipal Group Co., Ltd, Guangzhou, Guangdong 410060, China; ^4^Guicheng Transportation Service Institute of Nanhai District Transportation Bureau, Foshan, Guangdong 528253, China; ^5^Guangzhou Municipal Engineering Design & Research Institute Co., Ltd, Guangzhou, Guangdong 510060, China

## Abstract

Urban interchange is the core hub connecting various regions, and it is of great significance for alleviating the problem of traffic congestion. In the process of urban interchange design, it is impossible to strictly control the traffic volume, interchange types, and standards by relying on traditional technologies. Smart transportation and big data are emerging technologies based on data, which can provide technical support for design and decision making. Based on this, this paper first uses smart transportation and big data technology to predict the traffic volume of Nancheng New District, so as to calculate the future development trend of the target area. Then, on the basis of traffic volume, the article uses smart transportation and big data technology to optimize the original urban interchange design scheme from the aspects of traffic capacity, safety, economic benefits, and environmental benefits. Finally, the article evaluates the optimized urban interchange scheme by means of comprehensive quantitative indicators and evaluation methods. Experiments show that the traffic capacity of the interchange on the outer ring road optimized by smart transportation and big data has increased to 72.6%, and the environmental coordination has increased from 45.2% to 55.2%. Moreover, the design aesthetics of the urban interchange after optimized design based on smart transportation and big data has increased to 65.9%. In addition, the comprehensive evaluation value of the urban interchange after optimization of smart transportation and big data reached 82.6. This fully shows that the optimal design of urban interchange based on the integration of smart transportation and big data can greatly improve the traffic capacity of urban roads.

## 1. Introduction

With the rapid economic development, interchange projects have taken root in various regions, which alleviated regional traffic problems to a certain extent. However, different from the plane crossing, the urban interchange not only needs to consider land occupation and investment but also needs to consider the transportation organization and structure of the area. However, it is often impossible to accurately predict the local traffic volume using traditional techniques and cannot provide the correct direction for the subsequent urban interchange design. Smart transportation and big data are the traffic information complex in the new era, which can integrate the information of various traffic subjects. Therefore, the integration of smart transportation and big data can provide data support for the design of urban interchange and help formulate a reasonable design scheme for urban interchange. At the same time, with the help of smart transportation and big data, relevant departments can predict the future traffic form in advance in the process of urban interoperability optimization design, and realize advance planning. In addition, the urban interchange design based on smart transportation and big data optimization can ensure the safety of regional traffic to the greatest extent.

Urban interchanges are of great significance for improving urban traffic efficiency and improving traffic problems. Franco-Pérez et al. [1] pointed out that in existing urban interchanges, lane assignments and existing elevated guide signs and lanes are often modified, resulting in temporary misalignment. So, he conducted a driving study using simulators to determine whether drivers would be affected by temporary misalignment of permanent guide signs, temporary guide signs, and route-shielding pavement signs in a lane change position [1]. Finley et al. [2] aimed to analyze whether lighting in urban road interchanges has an impact on driver behavior. So, he measured on-site lighting data at urban interchanges using a time-series algorithm and then explored correlations between road lighting variables and several safety surrogate variables. Finally, he also aimed to improve the current lighting design system, hoping to create a safer lighting environment for drivers [2]. Wakui et al. [3] pointed out that accessibility is very important for urban road interchange design. Therefore, based on the route information of the navigation map software, he proposed a new comprehensive travel model that can dynamically analyze the accessibility of urban road interchanges. In addition, he also used the proposed model to study the dynamic accessibility of Zhengzhou expressway entrances and exits, and analyzed the calculation results [3]. Cekaite [4] pointed out that figure theory can be used to represent real-time road conditions in urban road interchanges. Among them, the road intersection where the roads intersect and the driver is not allowed to change lanes can be represented as a two-color one-way connectivity map. In addition, he also studied the minimum number of bridges at interchanges based on combinatorics and topology [4]. Homchaudhuri et al. [5] proposed a new multifunctional road interchange model. In this model, all the interchanges have only two floors, and only the circulation does not intersect, so their capacity is not limited by the design. Most importantly, these interchanges allow people to easily access the interior of other venues [5]. The above experts and scholars have put forward valuable opinions on the development of urban road interchanges from various perspectives, but they did not combine the latest smart transportation and big data technology in the research process.

Smart transportation and big data have provided new opportunities for transportation decision making and management, which have also attracted many experts and scholars to explore. Montoya-Torres et al. [6] pointed out that vehicle networks have great potential to improve road safety and traffic efficiency. At the same time, he studied the causes of road accidents using real-time accident big data obtained from the Florida Department of Transportation. On this basis, he designed a real-time big data system using a linear regression model and a distributed random forest framework to predict accidents and congestion before they occur [6]. Xiang [7] pointed out that as the urban population continues to grow, the need for intelligent transportation systems is becoming more and more important. The article first reviews the relevant literature on big data analysis of intelligent transportation systems. Then, on the basis of previous work, the paper proposes a simple and complete big data analysis architecture for integrated intelligent transportation systems [7]. In order to solve various problems in road traffic, Li [8] proposed a new prediction system. In this system, he calculated the traffic density and average speed of each road segment, and then, through parallel data processing, he predicted the risk of vehicle accident in an instant way [8]. Gruson [9] pointed out that with the widespread application of intelligent transportation equipment such as smart cards and road deceleration devices, the collection of multisource traffic data is easier than ever. Based on this, he analyzed and excavated the regularity behind the traffic big data, and then re-optimized the architecture of the intelligent transportation system [9]. Kumar studied the model base framework of the urban intelligent transportation data platform. In the research process, he integrated the big data mining model of design model, traffic model, traffic thematic analysis, and multithematic analysis with the traffic simulation platform. It realizes the functions of traffic status recognition and traffic analysis, and provides data support for better decision making, planning, and urban traffic control [10]. The above experts and scholars have fully explored the application of smart transportation and big data in traffic information mining, but they have not put forward substantive suggestions for the design of urban road interchanges.

Based on the integration of smart transportation and big data, this paper re-optimizes the design of urban interchange, fully develops a new direction of interchange design, and realizes the upgrade of urban interchange. After the new ramp was added, the ramp capacity of the interchange was the largest, up to 86.2% year-on-year. In the four directions of southeast and northwest, the accessibility of the optimized interchange has the largest improvement in the east and south directions, with a year-on-year increase of 7.12% and 6.52%. In addition, both the original scheme and the optimized scheme have good convenience, and their quantitative indicators basically reach 7, which is at a good level. However, it is also found that in terms of driving comfort, the level of comfort of the interchange design scheme after big data and smart traffic optimization is higher, with a value of 7, which is at a good level. By contrast, the driving comfort index value of the original plan is 5, which is at a general level. This fully shows that the optimal design of urban interchange based on smart transportation and big data can effectively improve regional traffic capacity and driving comfort. At the same time, it further illustrates the importance of using smart transportation and big data to realize the optimal design of urban interchange.

## 2. Urban Interchange under the Integration of Smart Transportation and Big Data

### 2.1. City Interchange

Urban interchange is an important choke for connecting urban areas and other economic areas. With the development of economy, the level of economic development between regions has been continuously improved, which has put forward new requirements for urban road construction. The design of urban interchange can realize spatial separation and continuous discontinuous traffic flow on plane intersections [11]. The schematic figure of the urban road interchange is shown in Figure 1.

Although the urban interchange can relieve the huge traffic pressure for the city, there are still many serious problems in the actual design of the urban interchange [12]. First, the regional long-term traffic volume forecast is the first problem that is difficult for us. In the process of traffic volume forecasting, common methods often fail to achieve accurate forecasting, which lays a hidden danger for subsequent interchange selection. On the one hand, if the predicted traffic growth rate is slower than the actual traffic volume, the built interchange will not be able to meet the future traffic needs of the region, thus hindering the economic development of the region [13, 14]. On the other hand, if the predicted traffic volume is much higher than the actual traffic volume, the built interchange will be idle, resulting in a waste of resources. Moreover, in this case, the coordination between the city interchange and the surrounding environment will also be broken. Therefore, accurate prediction of regional traffic volume will be the core of urban interchange design.

Secondly, there are various types of interchanges, and at the same time, they are restricted by various factors. The cost and function of different interchange types are also different. Moreover, the technical maturity corresponding to different interchange types is often not the same, which brings challenges to the builders. Finally, in actual operation, various factors such as investment cost, land use layout, intersection road conditions, and regional ecology should be comprehensively considered to determine the optimal interchange type [14, 15]. However, the existing technology cannot integrate all the above factors, so how to integrate various factors in the design of the interchange will be another difficult problem encountered in the design of the interchange.

### 2.2. Smart Transportation and Big Data

Smart transportation is a transportation service system that integrates a variety of modern technologies. In the development process of smart transportation, its integration with big data is the trend of the times. On the one hand, smart transportation relies on modern information technology, such as the Internet of Things, cloud computing, artificial intelligence, automatic control, mobile Internet, and other technologies, so it inevitably has to interact with data. On the other hand, the need for intelligent transportation itself promotes the combination of the two [14]. In the development process of smart transportation, it relies more and more on the support of data, so its combination with big data is the result of the combined effect of internal and external factors.

In this environment, the integration of smart transportation and big data brings dawn to the design of interchangeable interchanges. When designing an interchange, the future traffic volume in the area is an important reference for determining the type of interchange. However, due to technical and other reasons, there is often a certain difference between the estimated and predicted traffic volume. With the help of smart transportation and big data technology, the traffic volume prediction method has been adjusted, and its mathematical expression is as follows:

(1) $$\begin{array}{c} Y=\beta +v_{\ell },\\ T_{\left(i,j\right)}^{n}=T^{n}\frac{{ℒ}_{C}}{N_{Ci}},\\ N_{Ci}=\frac{T^{n}}{\sum \left(\ell_{i}^{n}\left(N_{Ci}/N_{ei}^{n-1}\right)\right)}. \end{array}$$

In the above formula, *𝒴* represents the traffic volume in the area in previous years, and *β* represents the time parameter. On the basis of the data over the years, we set up an automatic growth factor of *𝒯*. After each iteration, the traffic distribution will be double-constrained by the random vector ℒ_*𝒞*_ and the import and export flow *𝒩*_*𝒞i*_, so as to obtain the final prediction result.

After the predicted traffic volume is obtained, the basic pattern of the interchange can be basically established. Next, the designed interchange model needs to be evaluated to test its effect in practical application.

The traffic capacity can accurately measure the effect of interchange design, and its mathematical expression is as follows:

(2) $$\begin{array}{c} W=\frac{{ℱ}_{i}f}{t}\frac{S^{j}}{u_{o}}. \end{array}$$

Among them, *𝒲* represents the actual traffic capacity in the interchange structure, *t* represents the traffic flow per unit time, and *𝒮*^*j*^ represents the actual running speed of the vehicle.

In the forecasting process of the above traffic volume, the integration of smart transportation and big data is becoming more and more close, and this also puts forward new requirements for the integration of data. In order to realize the homology and unification of the data in the urban interchange design, this paper quantifies the relevant subjective indicators in the interchange, and the quantification results are shown in Table 1.

The table assigns actual quantified values to several indicators in interoperable design, which further accelerates the convergence between smart transportation, big data, and interoperable interchange design. In the actual design and construction process, it is also required that the interchange structure can integrate economic benefits and environmental benefits. Therefore, according to the above quantitative result table, the data processing of these two indicators is carried out as

(3) $$\begin{array}{c} K=m+b_{n}+f_{e}. \end{array}$$

In the above formula, *𝒦* represents the coordination of economic benefits and environmental benefits, *f*_*e*_ represents the quantified value of economic benefits, and *m* represents the environmental impact of the interchange structure during construction.

Through a series of quantification, measurement, and prediction, the basic efficiency of the interchange structure can basically be determined, but the above indicators are scattered and extremely inconvenient to calculate, so they are sorted and synthesized.

(4) $$\begin{array}{c} D=A^{*}\times C^{T},\\ A^{*}=n*Y+\gamma *W+K_{n},\\ C^{T}=\frac{n*Y+\gamma *W+K_{n}}{n*m}. \end{array}$$

Among them, *𝒟* represents the final score and result of the interchange scheme, *𝒜*^*∗*^ represents the weighted summation of the above indicators, and *𝒞*^*𝒯*^ represents the average value of each score indicator. Based on this, this paper initially integrates smart transportation and big data into the whole process of urban interchange design. Next, this paper will optimize the design under the comprehensive guidance of smart transportation and big data technology.

### 2.3. Optimal Design of Interchange Based on Smart Transportation and Big Data

Urban interchange is an important hub connecting various economic regions of the city, and it is of great significance for promoting regional economic development. Nancheng New District is one of the new urban areas that have gradually developed in recent years. With the economic development, the interaction between the urban area and the outside world has become more frequent. It is connected to the North Ring Expressway in the north, the Municipal Expressway in the east; intersects with the outer ring of the new district in the west; and connects with the South Ring Road in the south [16, 17]. Among them, the north-south expressway has a total length of 40.095 kilometers. The whole line is designed according to the standard of two-way six-lane urban expressway. The estimated driving speed is 80 kilometers per hour. In this context, the establishment of an interchange can greatly ease the city's traffic pressure and further promote regional economic development.

In order to establish the type of interchange, this paper first studies the traffic carrying capacity of the inner and outer ring roads, in order to determine the level and scale of this interchange in the roads of Nancheng New District. The results of the traffic carrying capacity of the outer ring and inner ring are shown in Table 2.

Table 2 shows that the traffic carrying capacity of the outer ring road is significantly higher than that of the inner ring road. Among them, the maximum motor vehicle carrying capacity of the outer loop is 96,584, while the inner loop is only 56,970. Due to the weak participation of pedestrians in the interchange, the influence of pedestrians on the carrying capacity is not considered in this paper. On the basis of the above traffic carrying capacity, we can know that the urban interchange to be established in Nancheng New District has a higher grade in the urban road. Using the traditional traffic volume forecasting algorithm, Nancheng New District counts the traffic forecast volume of the target area in different turning directions, and the results are shown in Table 3.

Table 3 shows that the traffic volume of Nancheng New District varies significantly in all directions. Among them, the traffic flow on the south and east sides of the new district is significantly more, and the maximum traffic flow per unit time can reach 3251. And in the right turn and straight direction, the traffic flow on this section is even more huge, with a value of 7951.

According to the traffic carrying capacity and traditional traffic volume forecast, Nancheng New District has designed the basic scheme of the interchange. Among them, in order to adapt to the right-turn traffic volume, the right-turn ramp in the new district adopts a directional or semidirectional ramp [18]. Others turn less traffic and therefore use roundabouts. So far, Nancheng New District interchange has initially established an interchange plan with a combination of left circular and right semidirectional.

Although Nancheng New District has carried out detailed traffic carrying capacity and directional traffic volume predictions for the destination, the predicted values are biased to a certain extent due to technical reasons. Moreover, in the design process, the new district did not take into account factors such as the safety of interchange driving. Therefore, on the basis of the traffic carrying capacity of part of the ring road in the new area, the traffic volume in this area is predicted by combining smart traffic and big data technology [19]. Among them, the forecast situation of the unit time flow of the destination is shown in Figure 2. According to the predicted traffic volume, it can be known that the traffic volume of the North Ring Road and the East Municipal Expressway is the largest, followed by the traffic volume of the South Ring Road.

Moreover, from the above forecast results of flow per unit time, we can also know that there are obvious tidal characteristics in the amount of vehicles on the east and south sides. This shows that for the prime time period, there will be a lot of traffic flow in the east and south loops of the Nancheng New District interchange [20]. The predicted traffic volume based on smart transportation and big data is shown in Table 4.

The predicted traffic volume in the area in the next 20 years is more representative of the future development of the area. Table 4 shows that based on big data and smart transportation, the traffic flow on the south and east sides of Nancheng New Area occupies the majority of the area. Its traffic flow per unit time can reach up to 4123. In the right turn and straight direction, the traffic flow on this section is even more alarming, and the value once rose to 8912.

Based on the above traffic volume forecast and flow forecast, on the basis of the original plan, an up-ramp was added in the south and east directions, and then also changed one of the roundabouts on the left to a semidirectional ramp. At the same time, the radius of the ramp has also been redesigned. On the one hand, this can reduce the stacking of on-ramps and interchange roundabouts. On the other hand, this can also ease the traffic flow during the prime time and reduce safety accidents.

## 3. Urban Interchange Optimization Results

The design of urban interchange is a very complex and comprehensive project, therefore, in order to compare the different schemes of the new district interchange design and verify the interchange optimization effect based on smart transportation and big data. The relevant data were quantified using the index quantification table designed. Among them, the comfort comparison results of the original scheme and the optimized scheme are shown in Table 5.

The data show that both the original scheme and the optimized scheme have good convenience, and their quantitative indicators have basically reached 7, which is at a good level. However, it is also found that in terms of driving comfort, the comfort level of the optimized solution based on big data and smart transportation is higher, with a value of 7, which is at a good level. By contrast, the driving comfort index value of the original plan is 5, which is at a general level. The reason is that the interchange design that integrates big data and smart transportation can take into account safety benefits while ensuring driving comfort.

In the process of studying the driving comfort, it is found that the traffic capacity will also affect the driving comfort. Therefore, it is also necessary to evaluate the traffic capacity of the interchange before and after optimization. The comparison results of urban interchange traffic capacity are shown in the table.

Table 6 shows that the traffic capacity of the urban interchange based on smart transportation and big data optimization is significantly improved. Among them, the traffic capacity of the optimized urban interchange on the ramp is improved from the original 5820 puc/h to 6230 puc/h, which greatly ensures the smoothness of the road on the ramp. Secondly, the traffic capacity of the optimized urban interchange on the main road reaches 7520 puc/h, and the traffic capacity on the ring road also reaches 6900 puc/h. This fully shows that the urban interchange design based on smart transportation and big data fully taps the traffic volume of each road and greatly improves the commuting efficiency of urban roads.

For the rationality of representation and the accuracy of the quantification process, the comfort quantification evaluation index table used in this paper will also be applicable to the quantification of economic benefits and environmental benefits. On this basis, the urban interchange is comprehensively optimized based on smart transportation and big data. The quantitative results of economic and environmental benefits before and after optimization are shown in Table 7.

Table 7 shows that the urban interchange optimized by the integration of smart transportation and big data is different from the original plan in terms of environmental and economic benefits. Among them, in terms of the coordination of the surrounding environment, the quantization value of the optimized design reaches 8, while the value of the original scheme is only 6. However, it was also found that the optimized design scheme increased the floor space to a certain extent, and its value increased from the original 77,000 square kilometers to 79,000 square kilometers. In this case, the cost of the optimized solution has also increased from 50.09 million yuan to 52 million yuan.

### 3.1. Urban Interchange Optimization Results

In the above, the intelligent transportation and big data are used to optimize the design of the interchange in Nancheng New District. But just relying on the above quantitative results cannot intuitively explain the pros and cons between the original scheme and the optimized scheme. Therefore, the above-mentioned evaluation method can be used to comprehensively evaluate the interchange scheme before and after optimization. The next article will explore the actual benefits of the two schemes one by one, starting from the traffic capacity, economic benefits, safety, and environmental benefits.

Deconstruction of the Optimized Urban Intercity Traffic Capacity: traffic capacity can accurately measure the actual performance of urban interchanges, and it is the basic index for evaluating the state of interchanges. Therefore, this paper compares the traffic capacity of the two schemes before and after optimization based on smart transportation and big data. The comparison results are shown in Figure 3.

Figure 3 shows that the traffic capacity of the optimized urban interchange has been greatly improved. Among them, the traffic capacity of the optimized interchange on the outer ring road increased to 72.6%, and the traffic capacity on the inner ring road increased to 73.8%. In addition, the optimized municipal express traffic capacity has been increased to 78.6%. In particular, after adding the new ramp, the ramp capacity of the interchange has the largest increase, up to 86.2% year-on-year. In the four directions of southeast and northwest, the accessibility of the optimized interchange has the largest improvement in the east and south directions, with a year-on-year increase of 7.12% and 6.52%.

Deconstruction of Economic Benefit of Optimized Urban Interchange: in the design process of urban interchange, economic benefits are the foundation of the project. In the design process, we should try our best to minimize the input economic cost and maximize the output economic benefit. At the same time, for the input cost, it is also hoped that it can be transferable. Among them, the comparison results of economic benefits between the optimization scheme based on smart transportation and the support of big data and the original scheme are shown in Figure 4.

Figure 4 shows that the difference between the economic benefits of interchange design before and after optimization is not very significant. Among them, in terms of project cost, the cost of the optimized plan is 33.12 million yuan, and the original plan is 33.21 million yuan, and the difference between the two is not significant. In addition, in terms of income, the basic income of the original plan is about 5%, and the basic income of the optimized plan is about 7%. In terms of the demolition area, the maximum demolition area of the original interchange design scheme is 3435 square kilometers, and the optimized maximum demolition area is 3521 square kilometers. The reason is that the optimized plan adds an up-ramp, which increases the cost of construction and expands the demolition area, but it also brings greater economic benefits.

Optimized Urban Interchange Safety Deconstruction: in the design process of the interchange, safety is the red line that cannot be touched by the design. Based on smart transportation and big data, the local safety accident situation is comprehensively analyzed, and then, a comprehensive analysis is carried out based on this. On this basis, the design of the interchange involving safety issues is re-optimized. The comparison of the safety of urban interchange before and after optimization is shown in Figure 5.

Figure 5 shows that the optimized design of the interchange greatly ensures the safety during driving. Among them, although the maximum allowable speed of the optimized interchange has increased from 100.3 kilometers per hour to 120.3 kilometers per hour, it has greatly shortened the commuting time and reduced unnecessary safety accidents. Moreover, in order to improve the safety of vehicles on the ramp, this paper re-optimizes the turning radius of the ramp, increasing the turning radius from the original 92 meters to 98 meters. The reason is that the traffic carrying capacity of the south and east sides is significantly larger than that of the other two directions. Therefore, increasing the turning radius of the ramp can better adapt to different traffic volumes and ensure smooth and safe roads.

Deconstruction of Environmental Benefits of Optimized Urban Interchanges: in the design process of urban interchange, environmental benefits are also an important factor to be considered. In the actual design process, the environmental friendliness of the urban interchange is an important reference to measure its future development. The environmental benefits of urban interchange before and after optimization are shown in Figure 6.

Figure 6 shows that the optimized urban interchange design has better environmental benefits. Among them, the environmental coordination of the optimized solution has increased from 45.2% to 55.2%, a year-on-year increase of 10%. Moreover, the aesthetics of the interchange design has increased to 65.9% after the optimized design based on smart transportation and big data. In addition, compared with the solution before optimization, the environmental friendliness of the urban interchange after optimization based on smart transportation and big data has comprehensively increased to 69.58%. The reason is that based on smart transportation and big data, the site can be selected comprehensively, and then, the urban interchange design can be carried out under the condition of ensuring coordination with the surrounding environment.

Based on the above, the urban interchange design scheme based on smart transportation and big data has a certain improvement in traffic capacity, economic benefits, safety, and environmental benefits. Combining with the comprehensive evaluation algorithm, we can further know that the final evaluation value of the original urban interchange is 81.4. The final evaluation value of the urban interchange after optimization of smart transportation and big data is 82.6. This fully shows that the integration of smart transportation and big data can reduce unnecessary economic investment in the construction of urban interchanges and reduce investment costs. At the same time, on the basis of alleviating urban traffic problems, urban interchange design based on the integration of smart traffic and big data can also comprehensively improve the social and economic benefits of urban road interchanges.

## 4. Conclusion

This paper takes the construction of the interchange in Nancheng New District as the main research object and focuses on the rationality of the implementation of the interchange scheme based on big data and smart traffic optimization. In addition, the paper conducts research from four aspects of traffic capacity, safety, economic, and environmental benefits and fully analyzes the actual benefits of the optimized interchange design scheme. Finally, the paper also uses a comprehensive evaluation method to evaluate the design scheme of the interchange before and after optimization. Experiments show that the optimal design of urban interchange based on smart transportation and big data can greatly improve the road capacity, safety, economic, and environmental benefits of Nancheng New District. In the actual design of interchangeable interchanges, the scheme design must be more than the above four points. However, due to time and other reasons, the article only optimizes the above four aspects. In the future, the article will comprehensively consider from multiple perspectives to obtain the optimal interchange design scheme.

## Figures and Tables

**Figure 1:** Schematic figure of urban road interchange.

**Figure 2:** Prediction map of target traffic per unit time.

**Figure 3:** Comparison of the capacity of urban interchange before and after optimization.

**Figure 4:** Comparison of economic benefits of urban interchange before and after optimization.

**Figure 5:** Comparison of the safety of urban interchange before and after optimization.

**Figure 6:** Comparison of environmental benefits of urban interchange before and after optimization.

**Table 1:** Indicator quantification results.

Grade	Numerical values
Very good	9
Good	7
General	5
Poor	3

**Table 2:** Outer ring and inner ring traffic capacity.

Road name	Outer ring road	Inner ring road
Motor vehicles	96584	56970
Pedestrians	12	20
Natural vehicles	26820	15820

**Table 3:** Predicted traffic volume in all directions at the destination.

Roads	2015		2025		2035	
	Left turn	Right turn	Left turn	Right turn	Left turn	Right turn
North side	2221	7548	2536	10121	3241	13210
South side	3030	7951	3681	12101	3520	13214
East side	3251	7254	3998	13410	3360	16213
West side	2581	7321	3021	16310	3421	15210

**Table 4:** Traffic volume forecast based on smart transportation and big data.

Roads	2020		2030		2040	
	Left turn	Right turn	Left turn	Right turn	Left turn	Right turn
North side	2229	8136	2698	13652	3321	17354
South side	4123	8912	3691	13214	3436	19962
East side	3131	8254	4031	16321	3698	19932
West side	2512	6325	3221	14369	3962	16360

**Table 5:** The comfort comparison results of the original scheme and the optimized scheme.

Related indicators	Comfort	Convenience	Security
Original program	5	7	6
Optimized solution	7	7	8
Average value	6	7	7

**Table 6:** Comparison results of urban interchange traffic capacity before and after optimization.

Related indicators	Ramps	Main roads	Expressways	Loop
Original program	5820	6830	6500	6720
Optimized solution	6230	7520	6830	6900
Average value	6025	7225	6615	6810

**Table 7:** Comparison of economic and environmental benefits.

Related indicators	Original program	Optimized solution	Average value
Surroundings	7	8	7.5
Aesthetics	6	8	7
Footprint	77000	79000	78000
Demolition area	6	6	6
Construction cost	5009	5200	5104.5

## Data Availability

The data used to support the findings of this study are available from the corresponding author upon request.
